The article "Hazard potential of volcanic flank collapses raised by new megatsunami evidence" was published in 2015. Journal: Sci Adv.

# Hazard potential of volcanic flank collapses raised by new megatsunami evidence

**DOI:** 10.1126/sciadv.1500456

**Published:** 2015-10-02

**Authors:** Ricardo S. Ramalho, Gisela Winckler, José Madeira, George R. Helffrich, Ana Hipólito, Rui Quartau, Katherine Adena, Joerg M. Schaefer

**Affiliations:** 1 School of Earth Sciences, University of Bristol, Wills Memorial Building, Queen’s Road, Bristol BS8 1RJ, UK.; 2 Lamont-Doherty Earth Observatory at Columbia University, Comer Geochemistry Building, 61 Route 9W, P. O. Box 1000, Palisades, NY 10964–8000, USA.; 3 Departamento de Geologia, Faculdade de Ciências, Universidade de Lisboa, 1749-016 Lisboa, Portugal.; 4 Instituto Dom Luiz, Faculdade de Ciências, Universidade de Lisboa, 1749-016 Lisboa, Portugal.; 5 Earth-Life Science Institute, Tokyo Institute of Technology, 2-12-1-IE-1 Ookayama, Meguro-ku, Tokyo 152-8550, Japan.; 6 Centro de Vulcanologia e Avaliação de Riscos Geológicos, Universidade dos Açores, Rua da Mãe de Deus, Edifício do Complexo Científico, 3° Andar–Ala Sul, 9500-321 Ponta Delgada, Açores, Portugal.; 7 Divisão de Geologia e Georecursos Marinhos, Instituto Português do Mar e da Atmosfera I.P., Rua C do Aeroporto, 1749-077 Lisboa, Portugal.

**Keywords:** volcanoes, Islands, geology, volcanic flank collapses, megatsunami, tsunami, natural hazard, Fogo, Santiago, Cape Verde Islands

## Abstract

Large-scale gravitational flank collapses of steep volcanic islands are hypothetically capable of triggering megatsunamis with highly catastrophic effects. Yet, evidence for the generation and impact of collapse-triggered megatsunamis and their high run-ups remains scarce or is highly controversial. Therefore, doubts remain on whether island flank failures truly generate enough volume flux to trigger giant tsunamis, leading to diverging opinions concerning the real hazard potential of such collapses. We show that one of the most prominent oceanic volcanoes on Earth—Fogo, in the Cape Verde Islands—catastrophically collapsed and triggered a megatsunami with devastating effects ~73,000 years ago. Our deductions are based on the recent discovery and cosmogenic ^3^He dating of tsunamigenic deposits found on nearby Santiago Island, which attest to the impact of this giant tsunami and document wave run-up heights exceeding 270 m. The evidence reported here implies that Fogo’s flank failure involved at least one fast and voluminous event that led to a giant tsunami, in contrast to what has been suggested before. Our observations therefore further demonstrate that flank collapses may indeed catastrophically happen and are capable of triggering tsunamis of enormous height and energy, adding to their hazard potential.

## Teaser

Giant tsunami triggered by catastrophic flank collapse of Fogo volcano.

## INTRODUCTION

The tsunamigenic potential of volcanic island gravitational flank collapses has long been recognized but remains poorly constrained (*1*–*4*). The lack of direct observations means that little is still known on the mechanics of collapse development, which play a fundamental role on tsunami generation (*2*–*4*). Additionally, onshore deposits documenting megatsunami (*5*) high run-ups are extremely rare (*6*, *7*) or are highly contentious (*8*–*12*), making the assessment of this geohazard even more problematic. In particular, doubts remain on whether large-scale flank failures typically result in highly devastating megatsunamis (*2*–*4*, *12*–*18*). At the center of the problem is the still largely unanswered question as to whether flank collapses generally happen catastrophically and generate enough volume flux to result in megatsunamis (*1*, *6*–*8*, *11*, *15*) or alternatively operate by slow-moving or multiple smaller episodic failures (*2*–*4*, *16*, *18*) with much lower tsunamigenic potential (*2*–*4*, *16*–*18*). Competent forecasting scenarios for the near- and far-field effects of collapse-generated tsunamis, however, hinge on this distinction.

Here, we focus on the Cape Verde archipelago off western Africa, where a massive flank collapse at Fogo volcano potentially triggered a giant tsunami with devastating effects, reportedly between 65,000 and 124,000 years ago (*17*, *19*, *20*). Fogo is one of the most active and prominent oceanic volcanoes on Earth, presently standing 2829 m above mean sea level and ~7 km above the surrounding seafloor. The island’s morphology is characterized by a young stratovolcano (Pico do Fogo) rising from a central depression that opens eastward. This depression has been interpreted as an old summit caldera (*21*), whose eastern flank failed and collapsed onto the sea (*17*, *19*–*23*), a deduction that is supported by the presence of submarine debris avalanche deposits extending offshore (Fig. 1). Analysis of swath bathymetry and backscatter data from the seafloor off Fogo delineates the offshore extension of a large field of avalanche debris, comprising a dislocated volume of 130 to 160 km^3^ of rock (*22*, *23*) (Fig. 1). If deposited in a single catastrophic event, a large tsunami may have ensued that affected the other Cape Verde Islands (*17*).

**Fig. 1:** Onshore and offshore evidence for Fogo’s flank collapse. Fogo’s flank collapse is documented by collapse scars onshore and by an avalanche debris field extending offshore, as illustrated in this digital elevation map of Fogo and Santiago and the surrounding seafloor (*22*, *23*). The study area on northern Santiago is marked with a rectangle, and the blue dots represent the general location of the tsunamigenic deposits reported in this study. The event timeline at the top compares the age interval previously suggested for Fogo flank collapse [in red (*17*–*19*)] with the depositional age interval for Santiago’s tsunamigenic deposits obtained in this study (blue). Topography of Fogo and Santiago corresponds to digital elevation model at 1:5000 scale (*31*, *32*). Seafloor mosaic is composed of low-resolution bathymetry [30 arc-second interval grid, (*33*)] and higher resolution bathymetry [200 m, (*22*, *23*)].

Our study concentrates on Santiago, an island that would have faced the worst effects of a giant tsunami originating at Fogo, being located just 55 km immediately offshore the collapse site (Fig. 1). Additionally, Santiago offers the unique advantage that its uplift trend is well constrained by independent sea-level tracers (*24*, *25*), minimizing the effects of relative sea-level uncertainties in wave run-up estimates. Tsunamigenic conglomerates linked to Fogo’s collapse have previously been reported at Tarrafal Bay in the NW coast of the island, but their location at low elevations (<15 m above the present sea level) precluded any reasonable wave run-up estimates (*17*).

## RESULTS

Our search for tsunamigenic deposits on Santiago included a high plateau bounded by vertical cliffs and lower concave slopes on the island’s northern tip. This plateau features large fields of boulders stranded on its smooth surface and chaotic conglomerates “plastered” against the adjacent lower slopes (Figs. 2 and 3, A to C). The large boulders (1 to 8 m in diameter, weighing 1 to 700 Mg) are particularly abundant around two sectors adjacent to the eastern banks of the northwest-oriented canyons of Ribeira Funda and Ribeira da Furna. In these two areas, the boulders occur scattered (with some clustering) from near the cliff edge at 160 to 190 m in elevation, up to ~220 m in elevation and 650 m inland. Several key characteristics suggest a tsunamigenic origin for these boulders (Fig. 3, A and B). First, they all correspond to blocks of basaltic submarine sheet flows (85%), fossiliferous limestones (11%), marine conglomerates (2%), or mafic tuffs (2%), which are lithologies that exclusively crop out on the cliff faces and lower slopes of the plateau, implying a source at considerably lower elevations. Second, all these boulders are stranded on top of young subaerial lavas that form the plateau’s surface, confirming their allochthonous origin. Third, the closer the source rock types on the cliff face are to the top, the more boulders of that lithology are on the plateau. This supports the scenario that the cliff edge itself was the source for most of the boulders. Effectively, most of the boulders correspond to the same submarine sheet flows that are exposed at the cliff edge, which frequently form protruding ledges as a result of differential erosion (Fig. 3D). This condition, together with the characteristic columnar and entablature jointing of these flows, would have facilitated the mechanical removal of joint-bounded large blocks by an incoming wave, thus explaining the relative abundance of boulders of this lithology over the plateau. Thus, taking into account the aforementioned characteristics, we infer that these boulders correspond to megaclasts that were quarried from the cliff edge and face (or eventually picked from the lower slopes if previously detached by downslope movement) and were transported uphill and inland onto the surface of the plateau. Only an exceptionally powerful tsunami would be capable of this upward and inland transport, making these the first tsunamigenic cliff-top boulder deposits known to date (*26*).

**Fig. 2:** Map of megatsunami field evidence on northern Santiago. Locations of large megaclasts are marked with dots, whereas chaotic conglomerates and sand sheets are mapped in pink. Contour line interval of 50 m. Rib^a^ Funda, Ribeira Funda; Rib^a^ da Furna, Ribeira da Furna. Topographic base: digital elevation model of Santiago Island, at 1:5000 scale (*32*).

**Fig. 3:** Megatsunami field evidence in northern Santiago. (**A**) Photos of tsunami megaclasts stranded on the surface of the plateau. (**B**) Schematic cross section of the NW slope showing the position of megaclasts and tsunamigenic conglomerates and sand sheets as well as the position of source rocks. (**C**) Photo of tsunamigenic conglomerates resting unconformably over friable carbonatites. (**D**) Photo of cliff face showing the protruding ledges of submarine flows that constituted the source for most megaclasts.

We applied cosmogenic ^3^He dating on the top surface of eight of the tsunami megaclasts. The ages of individual megaclasts range from 65 to 98 thousand years (ky), with the oldest age (TSU28) being an outlier within the 2σ level, which we exclude (fig. S1). The remaining seven ^3^He megaclast ages show fairly high internal consistency ranging from 65 to 84 ky, with an arithmetic mean of 73 ± 7 ky. Therefore, these results (see Materials and Methods) suggest a depositional age interval between 65 and 84 ky, with a more probable deposition age of about 73 ky (figs. S1 and S2). This timing is in agreement with the age interval of 65 to 124 ky previously suggested for Fogo’s flank failure (*17*, *19*, *20*), thus establishing the temporal link between a sudden tsunamigenic flank collapse at Fogo and Santiago’s tsunami deposits.

The impact of a megatsunami on Santiago’s shores is further supported by the occurrence of chaotic conglomerates and biocalcarenite sand sheets at lower elevations (Figs. 2 and 3C and fig. S3). These sediments cover the northwestern slopes (as steep as 20°) from near sea level up to ~100 m in elevation, resting directly on soils and friable carbonatites. Their maximum thickness amounts to 4 m, and they exhibit landward (and upslope) thinning and less pronounced fining. Sequences typically comprise one to three diffuse layers of extremely poorly sorted matrix-supported conglomerates often exhibiting landward imbrication, followed by sand sheets that form the topmost layer and may reach up to 1.5 m thick. These characteristics indicate tsunamigenic inland deposition, an observation also consistent with the conglomerates’ chaotic texture, featuring the typical mixing between marine and terrestrial materials (including rip-up clasts of friable tuff). Furthermore, the extreme heterometric composition of the conglomerates—with clasts ranging from a few centimeters up to 4 m in diameter—also implies an exceptionally energetic depositional process, possibly involving a combination of bed load and suspended transport modes as suggested for other tsunami deposits (*27*, *28*).

Several key observations point to a west-approaching tsunami that refracted around the northern coast of Santiago, caused catastrophic flooding of the northwest-oriented valleys, and subsequently spilled over the plateau (Fig. 4). This scenario is consistent with an event originating at Fogo and is supported by the spatial distribution of Santiago’s tsunamigenic deposits. This distribution reflects a preferential deposition of megaclasts, conglomerates, and sand sheets on either the eastern banks of the northwest-oriented canyons or the northwestern lower slopes, implying a main transport direction toward the eastern quadrant. Effectively, more than 90% of the megaclasts stranded on the plateau are located between 100 and 650 m inland from the cliff edge at the eastern bank of both Ribeira Funda and Ribeira da Furna, with most of the larger megaclasts closer to this feature. This suggests a transport direction toward SE or ESE, which is also compatible with the megaclasts’ long-axis orientation. Observations on historical tsunami deposits suggest that the megaclasts’ long-axis orientation tends to be approximately perpendicular to the direction of the tsunami flow (*27*, *28*); in this case, these orientations are generally oblique or quasi-perpendicular to the valley axis or the slope dip for megaclasts distant from valley walls, in agreement with the inferred flow direction (Fig. 4). Furthermore, catastrophic flooding of the valley of Ribeira Funda involving intense upstream knickpoint erosion is attested by the presence of a cluster of very large megaclasts and remains of biocalcarenite sand sheets in its upper reaches, above a prominent waterfall (Fig. 4 and figs. S4 and S5).

**Fig. 4:** Megaclast spatial distribution and interpreted tsunami inundation pattern. (**A**) Megaclast distribution by lithology, showing possible source regions (in red) and inferred transport direction when source areas are restricted enough to allow this interpretation (black arrows). Close-ups of regions 1 and 2 represent megaclast distribution by mass (in megagrams) and long-axis orientation. (**B**) Interpreted tsunami inundation pattern denoting a western-approaching tsunami that refracted along Santiago’s northern shore, caused flooding of the northwest-oriented valleys, and subsequently spilled over the plateau. Topographic base: digital elevation model of Santiago Island, at 1:5000 scale (*32*).

On the basis of the maximum elevation at which the tsunami megaclasts occur (220 m), we estimate a wave run-up in excess of 270 m, assuming coeval eustatic sea level (*29*) at −60 m and an uplift rate of 0.1 m/ky (*24*, *25*) (see Materials and Methods). Our estimations are minimally affected by relative sea-level uncertainties, because these probably amount to no more than 10% of the elevation at which the megaclasts occur. Our calculations of the upward flow rate channeled by the canyon geometry needed to raise the largest megaclast above the cliff edge (see Materials and Methods for details) implies a minimum incoming wave height of 170 m at the coeval shoreline. These characteristics make this event one of the largest megatsunamis preserved in the geological record (*17*).

## DISCUSSION

Previous studies reported that the tsunamigenic conglomerates found at Tarrafal Bay show evidence of at least two waves with successive inflow and outflow (*17*). These characteristics led to the suggestion that Fogo’s flank collapse possibly involved successive small retrogressive failures rather than a single massive event and did not generate a megatsunami (*17*). Our observations, however, require a megatsunami resulting from Fogo’s flank collapse, being in better agreement with numerical simulations that assume a single fast and coherent failure event scenario (*17*). Therefore, when integrated with observations from Tarrafal, our new evidence portrays a sequence of events in which a massive, sudden initial collapse led to smaller retrogressive events, resulting in an initial colossal wave followed by smaller replicas. Such a scenario would also result in distal multiphase collapse-related turbidite sequences, a feature observed offshore other collapse sites (*2*, *3*, *16*) and often suggested as evidence against megatsunami generation by just a single fast collapse.

We showed here that a massive tsunami affected the coastline of Santiago Island 73,000 years ago, and we have established the link with its source: a giant flank collapse at Fogo volcano. Our observations provide another line of evidence that large-scale flank failures at steep volcanic islands may indeed catastrophically happen and are capable of generating megatsunamis with devastating near-source effects. This new evidence therefore reinforces the hazard potential of volcanic island collapses and stands as a warning that such hazard should not be underestimated, particularly in areas where volcanic island edifices are close to other islands or to highly populated continental margins, such as in the NE Atlantic. In our opinion, the discussion should now focus on understanding the physics of flank collapses and their trigger mechanisms and on megatsunami generation, propagation, and inundation. Additionally, we should improve our knowledge on the far-field effects of collapse-generated waves. Unlike earthquakes, flank collapses essentially generate point-sourced tsunamis that lose intensity faster as their effects propagate to the far field (*14*, *30*). However, numerical models are still uncertain in their details of far-field effects, which depend on complex patterns of dispersion, refraction, and interference in wave propagation, as well as the parameters of the collapse source (*14*, *30*). Further research is therefore needed to address these questions. Only then, with a better understanding of the near- and far-field effects of collapse-generated megatsunamis, are we able to realistically assess the full hazard potential of such low-probability but high-impact events.

## MATERIALS AND METHODS

### Boulder morphometrics

We calculated megaclast volumes by approximating their shape to that of a prism, that is, volume = *l* × *w* × *h*. Masses were calculated using ρ_(basalt)_ = 2900 kg/m^3^, ρ_(limestone)_ and ρ_(conglomerate)_ = 2300 kg/m^3^, and ρ_(mafic tuff)_ = 2800 kg/m^3^. Megaclasts smaller than ~0.5 m^3^ were not considered in this study. The position of each megaclast was determined with a handheld Global Positioning System with a typical error of ±5 m. Megaclast long-axis orientation is given relative to geographic north and was only considered when this dimension was at least 30% longer than the nearest other dimension.

During the course of our study, we identified a total of 44 megaclasts (larger than ~1 m^3^), which are unambiguously stranded on the surface of the plateau in northern Santiago. In all cases, a downslope origin (hence upslope transport) could be easily asserted. In addition, at Baía de Angra—an enclosed bay on the eastern side of the area—five other large boulders were identified as tsunami megaclasts because their origin could be unambiguously assigned to marine sediment outcrops (conglomerates) located downslope of their present location, along the southern coast of that bay. Therefore, a total of 49 megaclasts were recorded in the area comprehended by this study (large boulders included as clasts within the conglomeratic deposits are not being considered for these statistics, as are any boulders found on the concave slopes whose downslope origin could not be safely inferred). From these 49 megaclasts, most correspond to basaltic submarine sheet flows, which exhibit the very distinctive columnar and entablature jointing typical of this lithology (see Fig. 2). These characteristics greatly contrast with the subaerial lava flows where the boulders rest, which generally exhibit the typical slab jointing of subaerial sequences. Moreover, because these boulders are often elongated according to the prisms’ long axis, their columnar jointing is often quasi-parallel to the topographical surface where they rest; this disposition is in contrast to the quasi-vertical position of the prisms found in in situ outcrops of submarine sheet flows exposed along the cliff face and serves to attest their nature as megaclasts stranded on the surface of the plateau. In a similar fashion, all other types of megaclasts correspond to lithologies that are unambiguously—and exclusively—exposed along the cliff face and lower slopes, further attesting to a downslope origin.

A careful analysis on the distribution of megaclasts along the plateau reveals that more than 90% of them are located between 100 and 650 m inland from the cliff edge at the eastern bank of both Ribeira Funda and Ribeira da Furna, at elevations ranging from 146 to 220 m above the present sea level (with 98% of the megaclasts above 160 m). The megaclasts are generally scattered along the plateau’s surface but sometimes form clusters, some of which correspond to a larger boulder that was broken into smaller clasts upon deposition (see Fig. 3A, central and central-right subfigures). In terms of their mass, the megaclasts range from ~1 to ~700 Mg. However, most of the megaclasts exhibiting a mass in excess of 150 Mg are clustered in the upper reaches of Ribeira Funda, above a prominent knickpoint (see Fig. 4 and fig. S4). The boulder located at the highest elevation (220 m) exhibits a mass of ~16 Mg and can be found ~240 m inland of the cliff edge (15°19′4.73″N, 23°41′56.62″W). In terms of long-axis orientation, all elongated boulders typically rest with their elongation oblique or quasi-perpendicular to the valley axes, or quasi-perpendicular to the slope dip for megaclasts distant from the cliff edges, a situation that is particularly evident at Achada Costa (see region 2 of Fig. 4A).

The aforementioned characteristics, in our opinion, can only be explained by tsunami upward and landward transport, toward the eastern quadrant, that is, with a tsunami wave (or train of waves) approaching from the west, refracting clockwise around the northern tip of the island, and resulting in extreme valley flooding and consequent spilling over the plateau. This transport direction would explain the preferential deposition of megaclasts on the eastern banks of the canyons, their general distribution on the area, and the preferential deposition of conglomerates on the western and northwestern lower slopes. In a similar fashion, it would explain the megaclasts’ preferential long-axis orientation, because evidence from historical tsunamis (*27*, *28*) suggests this direction to be roughly perpendicular to tsunami flow direction. The inferred clockwise refraction of the wave is also supported by field evidence. On the western side of Achada Bilim (region 1 in Fig. 4A), a lone megaclast weighing 185 Mg is presently located at 215 m in elevation, yet its origin can be placed 600 m to the SW, at the cliff edge (this origin is inferred on the basis of its very distinctive columnar jointing, which only occurs in outcrops exposed in that part of the cliff). This transport direction is therefore compatible with an incoming wave from the WSW, in the SW part of the area. In contrast, further north, the megaclast distribution suggests a transport toward the SE or ESE, which resulted in valley flooding. In this area, the cluster of very large megaclasts above the waterfall at Ribeira Funda, in our opinion, constitutes as evidence for catastrophic valley flooding, leading to extreme upstream knickpoint erosion and consequent deposition above this point, further attesting to this transport direction. Finally, at Baía de Angra, megaclasts (ranging from 11 to 54 Mg) presently located at ~30 m in elevation can be unambiguously traced back to their source outcrops located ~300 m to the SSE and 25 m lower, suggesting transport from the SE. This transport direction would be compatible with a tsunami that wrapped around the northern tip of the island and propagated southward along the eastern coast, bouncing on the southern coast of the bay.

### ^3^He chronology

We collected samples from the top surface of selected megaclasts using hammer and chisel, for ^3^He cosmogenic dating. We focused on the center of the megaclast’s upper surface and on areas without obvious erosion, that is, where the faces of the columnar-jointing prisms were preserved and retained the typical weathering patina. Sampled lithologies correspond to quenched submarine basalts with abundant olivine phenocrysts <200 μm and rare 200-μm to 1-mm olivine phenocrysts. High-purity olivine separates were extracted from crushed samples (using only the upper 3 to 5 cm) by density and magnetic separation techniques and subsequent leaching in 2% hydrofluoric/nitric acid on the shaker table for 2 hours. Average grain fraction ranged from 63 to 125 μm.

Mineral separation and helium isotope analyses were performed at Lamont-Doherty Earth Observatory of Columbia University. Eight samples were analyzed for helium isotopes after complete extraction in a furnace, and one sample was analyzed after in-vacuum crushing. For the total extractions, about 200 mg of olivine separates was wrapped in aluminum foil and degassed in vacuum in a molybdenum crucible at ~1300°C, using a resistance-heated double-walled furnace. For the magmatic He test, we extensively crushed about 0.5 g of mineral grains under vacuum with an automated piston for three 60-piston cycles interrupted by a 10-min break to prevent overheating of the electromagnets. Extracted gas was purified by exposure to a liquid nitrogen–cooled cryogenic charcoal trap and a SAES getter and trapped at 15 K on activated charcoal in a cryogenic absorber; helium was separated from the neon fraction at 45 K before it was inlet and analyzed in a MAP (Mass Analyzer Products) 215-50 noble gas mass spectrometer by peak jumping (*34*, *35*). ^4^He and ^3^He concentrations were calibrated against a 0.1-cm^3^ pipette of our standard gas (Murdering Mudpot) with an elevated ^3^He/^4^He ratio of 16.45 Ra. Standard reproducibility during the period of the measurements was ~1% (1σ) and ~1.5% (1σ) for ^4^He and ^3^He, respectively. In addition to the reproducibility of the calibration standard gas, the reported uncertainties include internal measurement precision, uncertainty associated with the nonlinearity correction, and the uncertainty in the blank subtraction. Hot blanks were measured for every crucible and yielded 0.1 to 0.2 ncc STP of ^4^He with atmospheric isotopic composition and blank corrections representing <1% of ^4^He for most of the samples.

To calculate ^3^He exposure ages from the measured total ^3^He concentrations (table S1), we considered the potential contribution of magmatic helium [for example, (*36*, *37*)] as well as the ^3^He produced by thermal neutrons via the ^6^Li(n,α)^3^H(β)^3^He reaction (*38*). All our mineral separates were aggressively leached in hydrofluoric and nitric acid, successfully dissolving the outer rims of the 63- to 125-μm mineral grains (*39*) and in turn substantially reducing the contribution of radiogenic helium implanted in the outer rims of our minerals by α-decay from U/Th-rich accessory minerals. Table S2 shows the inductively coupled plasma (ICP) analysis from splits of the mineral separates used for the helium analysis. Li concentrations in our mineral separates from lava flows 2.54 to 2.33 million years (*24*, *25*) in age are consistently low (~4 to 5 ppm); thus, the thermal neutron ^3^He component produced in situ in our minerals is low. We therefore consider the contribution of nucleogenic ^3^He to be negligible (*40*).

As for the magmatic helium control, we followed recently reviewed protocols (*36*) to minimize the contribution of magmatic helium. We used microphenocrysts of grain sizes <200 μm (*41*). Optical inspection of our minerals did not reveal any evidence for inclusions. We performed a prolonged in-vacuum crushing test for one of our mineral separates (TSU11-1, table S1), of about 200 mg of olivine, which should release all of the magmatic helium (*42*). This intensive crushing procedure yielded only a small amount of helium (~1% of the total ^3^He in the degassed olivine samples, see table S1). Although it is unclear whether this small helium component released by crushing is purely magmatic or a mixture of magmatic and radiogenic helium, we conclude that nearly all ^3^He is cosmogenic in origin. We estimated the radiogenic ^4^He production (*43*) in our samples since their extrusion at 2.54–2.33 million years ago on the basis of measured U and Th concentrations (table S2), and these theoretical values are consistent with the observed values (table S1). We therefore infer that practically all the ^4^He measured in these olivines is rediogenic. Accordingly, we base our ^3^He surface exposure age calculations on the ^3^He concentrations shown in table S1. Independent support for this argument is provided by the internal consistency of the ^3^He exposure ages, which is hard to explain if noncosmogenic ^3^He components were significant.

For the age calculations (table S3), we used the global ^3^He production rate compilation based on no- or low-erosion surfaces (*44*–*46*). We also considered the locally derived long-term ^3^He production rate (*47*), which is 15 to 20% lower than the global rate (*44*). However, we chose to not apply this local ^3^He production rate because the surfaces at the calibration site (*47*) show signs of erosion, thus potentially making this local ^3^He production rate inappropriate for the low-erosion boulder surfaces dated here. It is important to note, however, that the conclusions here presented do not depend on the choice between these two production rates. Free horizon parameters were measured in the field, using a sighting compass and clinometer, and correction for landscape shielding corresponds to 1% or less (see table S1).

Previous studies suggested a probable age for Fogo’s flank collapse, that is, about 65 to 124 ky (*20*) or, more recently, about 86 to 124 ky (*17*). The upper bound rests on both a single U-Th age (123 ± 3.9 ky) yielded by a piece of coral found within the conglomerates at Tarrafal Bay (*17*) (Santiago) and the exposure age (~123 ky) of a lava flow from Fogo interpreted as precollapse (*17*). The 86-ky lower bound, on the other hand, rests on a single K-Ar age (86 ± 3 ky) of a reportedly “postcollapse” lava flow from Bordeira (Fogo) (*17*). However, opinions diverge on whether this dramatic geomorphological feature (albeit eroded) represents the gravitational collapse headwall (*19*, *20*) or instead represents a volcanic caldera wall that predates the gravitational collapse (*21*, *48*–*50*) (fig. S6). The latter opinion is essentially based on two aspects: (i) the local morphology suggesting the presence of two semicircular “calderas” at slightly different elevations, which are assumed to correspond to two volcanic caldera-forming events, and (ii) the presence of a thick sequence of block and ash flow deposits intercalated within the Bordeira exposed volcanic succession, which may attest to at least one caldera-forming event (*21*, *48*–*50*). If these assumptions are correct, the 86 ± 3 ky age obtained from the Bordeira lava flow corresponds to the minimum age for the caldera-forming event(s) and not the minimum age for the gravitational collapse that postdates the caldera(s). Therefore, taking into account that it is still not entirely clear what the Bordeira wall represents, the 86-ky lower age bound previously suggested for Fogo’s flank failure must be considered with caution.

The tsunami depositional age interval reported here corresponds to 65 to 84 ky, with a mean at 73.3 ± 6.8 ky. These ages completely overlap with the previously suggested age interval of 65 to 124 ky (*20*) but not the age interval of 86 to 124 ky (*17*). This discrepancy is, in our opinion, related to the aforementioned problem. Therefore, we consider our ages to be consistent with Fogo’s flank collapse, eventually providing a more solid constraint on the timing of this event than previous estimates.

### Wave run-up and tsunami height calculations

We calculated wave run-up using the elevation of the highest megaclast at 220 m in relation to the coeval eustatic sea level (*29*) (averaged for the age interval) at −60 m and correcting for ~7 m of uplift since deposition (using an uplift rate of ~0.1 m/ky) (*24*, *25*), that is, 220 − (−60) − (+7) = 273 m.

Tsunami run-up is a complex process governed by local bathymetry and topography. Various authors made simplifying assumptions about these, leading to some successful and oft-cited formulae for run-up distance in, for example, planar geometry (*51*) and circular island geometry (*52*). The Santiago deposit presents three problems that thwart attempts to apply simplified system formulae: first, the topography is not even approximately planar through the megaclast deposition range; second, the topography varies laterally along the coastline; and third, the wavelength of the wave is not known.

Methods previously used to assess tsunami height from the positions and masses of transported boulders rely on relating transport factors (forces of lift, drag, and rolling) to incoming tsunami heights (*53*). Flow due to a lateral bore of constant depth is the initial approximation used or a variable-depth soliton-like wave whose peak-to-trough amplitude is a few tens of meters at most. These methods serve to provide a weak lower bound on wave height because they assume that the wave already overtops the levels at which the transported rocks lie. In the case of the Santiago deposit, the weak bound is 273 m.

Both the offshore bathymetric profile and the topography of Ribeira Funda have slopes of ~15°. Because simulations of solitary wave propagation in shoaling waters do not result in breaking over slopes greater than 12.5° (*54*), we do not need to consider water jet formation on impact of breaking waves on barriers, as did Cooker and Peregrine (*55*). In any case, barrier surface roughness, such as the uneven face of the canyon, apparently hinders jet development (*56*).

Consequently, we seek a treatment that uses the dominant factor of the flow related to the deposit: the physical lifting of the megaclast from its outcrop location to its position on the plateau. Because the outcrops are at or below the Ribeira Funda cliff edge, finding the megaclasts on top of the plateau puts a firm lower bound on the upward flux. The megaclast transport is due to entrainment in a turbulent flow (assumed, but likely); hence, we use the generic turbulent drag coefficient *C*_D_ = 0.5 and equate the body force of the megaclast to the drag force (*57*). Thus, the settling speed *v* is

$$v^{2}=\frac{8}{3}\frac{rg}{C_{D}}$$ (1)

where *r* is the radius of a spherical megaclast with the same mass and *g* is the gravitational acceleration. Using 700 Mg as the largest clast and a density of 2900 kg m^−3^, *r* is ~4 m, and thus the turbulent vertical flux must be >14 m s^−1^.

The dominant run-up factor is the narrowing topography of Ribeira Funda, whose shape in map view is approximately triangular (a recumbent triangular prism in three dimensions). A constant water flux into the ocean-facing rectangular base necessitates a rise in level due to inland narrowing of the valley and the reduction in cross-sectional area. We ask, when does the rate of rise equal the suspension velocity for a megaclast? Writing a relation for the mass flux *dM*

dM=ρA(l)dl (2)

where ρ is the water density, *A* is the area of inflow through the base, and *dl* is a differential flow length through *A*. We assume that water flows at a constant rate across the base, consistent with other models of tsunami effects that posit a constant depth bore or the average water flux of a soliton-like wave crossing the base (*53*). If the water mass is conserved once it crosses the shoreline, then

$$\frac{dM}{dt}=0=\rho A(l)c$$ (3)

where *c* is the speed of the incoming wave at the shoreline. Thus, for incompressible water and a constant *c*

$$\begin{array}{c} 0=\frac{d}{dt}[\rho cA(l)]\\ =\frac{d}{dt}[w(l)h(l)]\\ =w(l)\frac{dh(l)}{dt}+h(l)\frac{dw(l)}{dt}\\ =w(l)\frac{dh(l)}{dt}+h(l)c\frac{dw(l)}{dl} \end{array}$$ (4)

The area *A* depends on *l*, the distance above the base, through a functional dependence of the width *w* and height *h* on *l*. Specifically, *w* = *w*_0_(1 − *l*/*l*_0_) and *h* = *h*_0_(1 − *l*/*l*_0_), where *w*_0_ and *h*_0_ are the width and height of the base at the waterline, respectively, and *l*_0_ is the distance from the coeval shoreline to the cliff edge, which is ~1.5 km. Rearranging Eq. 4 and dropping the explicit dependence of *w* and *h* on *l*

$$w\frac{dh}{dt}=-ch\frac{dw}{dl}$$ (5)

and thus

$$\begin{array}{c} \frac{dh}{dt}=-c\frac{h}{w}\frac{dw}{dl}\\ =-c\frac{h_{0}(1-l/l_{0})}{w_{0}(1-l/l_{0})}\frac{-w_{0}}{l_{0}}\\ =c\frac{h_{0}}{l_{0}} \end{array}$$ (6)

Using Eq. 6 and *dh*/*dt* estimated above and the wave speed *c* = (*gd*)^1/2^ with an offshore water depth *d* of 1500 m and *g* = 9.81 m s^−2^, we get a minimum tsunami wave height of 170 m at the shoreline. This is approximately the level of the plateau on which the megaclasts sit and, post hoc, confirms the suitability of the approximations used.

The water depth here represents the average water depth on the slope of the immersed volcanic edifice (Fig. 1); ignorance of the wavelength of the incoming wave hampers any more refined choice. Because the tsunami wave height is linearly related to *c*, a factor of 2 variations in depth would lead to ±40% changes in height. Thus, the weak bound of ~270 m and the slightly stronger lower bound of 170 m indicate that the tsunami height is a substantial fraction of the plateau height. Simulation of collapse-generated tsunamis in the near field show waves of this height to be plausible (*17*, *58*).

### Tsunami conglomerates of northern Santiago

We describe here the conglomerates and sand sheets that, together with the megaclast fields of Achada Bilim and Achada Costa, document the impact of a megatsunami on the northern tip of Santiago. These sediments are particularly well represented in the northwestern lower slopes bordering Achada Bilim (see Fig. 2). In this area, the deposits rest on slopes dipping up to 20° and from the present sea level up to 100 m in elevation. They stand on the topographic surface, being preserved in interfluves between gullies incising the steep slopes (see fig. S3A). The base of the deposits is irregular, corresponding to an erosional surface cut on friable mafic and carbonatitic tuffs or tuffites but without an abutment unconformity (fig. S3, B to E).

The deposits are generally composed of one to three diffuse layers of extremely poorly sorted or chaotic conglomerates and sand sheets presenting a maximum thickness of 4 m. The sediments present landward (and upslope) thinning and less pronounced fining. The internal structure of the sedimentary sequence (that is, number, geometry, and nature of layers) rapidly changes both laterally and upslope from one outcrop to the other. However, a general fining upward sequence is present, with sand sheets typically comprising the topmost layer.

The texture of the conglomerates varies from matrix- to clast-supported. Matrix composition generally corresponds to medium-to-coarse bioclastic sandstone and is slightly lithified and calcretized. The dominant bioclasts are rhodolith fragments, but clasts of mollusks, coral, bryozoans, and foraminifers are also present, demonstrating a marine origin for the sand. In a similar fashion, featured macrofossils are marine in nature and include whole and broken rhodoliths, coral heads, bivalve and gastropod shells or shell fragments, and bryozoans. The fossil content and the amount of marine sand decrease landward, whereas the terrigenous contribution (angular clasts and colluvial sand) increases. The clasts in the conglomerates present both well-rounded (beach pebbles) and angular shapes and vary in size from 1 cm up to several meters (megaclasts). Frequently, the largest megaclasts are just partially buried by the conglomerate and sand sheets, with the top protruding above the surface of the topmost layer (fig. S3, A, B, C, and E). Locally, lenses of well-rounded pebbles can be found within the deposit, with landward imbrication. These are usually matrix- to clast-supported, embedded in a calcarenite matrix. Dominant clast lithology corresponds to dense basalt, sourced from the submarine sheet flows exposed at the cliff face. Angular clasts of marine limestone are also present (fig. S3F). Rounded pebbles are usually smaller than 25 cm in diameter, whereas angular and subangular clasts vary from a few centimeters up to several meters. The largest megaclasts of massive jointed submarine basalt range from 5 to 80 m^3^ in volume, corresponding to blocks weighing up to 220 to 240 Mg (see fig. S3, A, B, C, and E). These were probably detached from the cliff face by downslope movements and later picked up and incorporated within the conglomerates by the same depositional event.

The lower part of the sedimentary deposits contains occasional clasts of friable tuff up to 20 cm in diameter; these were eroded from the underlying basement and incorporated in the deposits as rip-up clasts (fig. S3D). In several locations, sand sheets are present, typically on the upper part of the sedimentary sequence (see Fig. 3 and fig. S3, A and E). These sand layers are dominantly bioclastic in nature, and the internal structure is massive or exhibits faint undulated stratification; dispersed clasts, both rounded and angular, are also abundant.

The aforementioned characteristics—deposition on top of steep slopes, erosional base, presence of fragile rip-up clasts, mixture of marine and terrestrial materials, mixture of rounded and angular clasts, marked structure variability, and so on—are all classic tsunamigenic characteristics (*6*–*8*, *17*, *27*, *59*, *60*). Therefore, we interpret these sediments as tsunamigenic in origin, in agreement with our interpretation on the origins of the fields of megaclasts.

## SUPPLEMENTARY MATERIALS

Supplementary material for this article is available at http://advances.sciencemag.org/cgi/content/full/1/9/e1500456/DC1 Fig. S1. Sample location and respective ^3^He cosmogenic ages around Ribeira Funda and Ribeira da Furna. Fig. S2. Normal kernel density estimate of ^3^He cosmogenic ages for sampled tsunami megaclasts. Fig. S3. Photos of tsunami sediments located on the lower northwestern slopes. Fig. S4. Knickpoint at Ribeira Funda. Fig. S5. Vestiges of tsunamigenic biocalcarenites at the upper reaches of Ribeira Funda. Fig. S6. Competing models concerning the origins of Bordeira. Table S1. ^3^He sample locations, geometrical corrections, and noble gas mass spectrometry from total extraction at ~1300°C and in-vacuum crushing. Table S2. ICP analysis from splits of the mineral separates used for the helium analysis. Table S3. ^3^He surface exposure ages of selected tsunami megaclasts.
